The article "How to Enhance Digital Support for Cross-Organisational Health Care Teams? A User-Based Explorative Study" was published in 2020. Journal: J Healthc Eng.

# How to Enhance Digital Support for Cross-Organisational Health Care Teams? A User-Based Explorative Study

**DOI:** 10.1155/2020/8824882

**Published:** 2020-09-15

**Authors:** Berglind F. Smaradottir, Gro K. Rosvold Berntsen, Rune W. Fensli

**Affiliations:** ^1^Department of Clinical Research, Sørlandet Hospital Trust, Post Box 416, Kristiansand N-4604, Norway; ^2^Department of Information and Communication Technology, University of Agder, Post Box 422, Kristiansand N-4604, Norway; ^3^Norwegian Centre for E-Health Research, University Hospital of North Norway, Post Box 35, Tromsø N-9038, Norway; ^4^Department of Community Medicine, The Arctic University of Norway, Post Box 6050 Langnes, Tromsø N-9037, Norway

## Abstract

Health care service provision of individualised treatment to an ageing population prone to chronic conditions and multimorbidities is threatened. There is a need for digitally supported care, that is, (1) person-centred, (2) integrated, and (3) proactive. The research project *3P*, *Patients and Professionals in Productive Teams*, aimed to validate and verify the prerequisites for health care systems run with patient-centred service models. This paper presents an explorative study of the digital support of a cross-organisational health care team in Norway, providing services to elderly frail people with multimorbidities in hospital discharge transition. Qualitative research methods were employed, with interviews and observations to map and evaluate the information flow and the digital support of collaborative work across organisations. The evaluation showed a lacking interoperability between the digital systems and a limited support for cross-organisational teamwork, causing raised manual efforts to maintain the information flow. Tools for coordination and planning across organisations were lacking. To enhance the situation, principles for a cloud-based health portal are proposed with a shared workspace, teamwork functionality for cross-organisational health care teams, and automatic back-end synchronisation of stored information. The main implications of this paper lie in the proposed principles which are transferable to a multitude of clinical contexts, where ad-hoc based access to shared medical information is of importance for decision-making and life-saving treatment.

## 1. Introduction

There is a need for innovative action to face the sharp increase of persons with multimorbidity and chronic conditions [1, 2], which threatens the sustainability of the health care systems [3–5]. This patient group dominates the 10% highest-care-spenders that utilise 2/3 of the care budget [6–8]. This group typically has multiple care processes, care providers, organisations, and care levels over longer periods of time. This puts frail multimorbid patients at documented risk for suboptimal care processes and outcomes, which in turn drives costs. However, health organisations tend to have an organisational fragmentation with a siloed structure, which also jeopardises the information flow [9]. Quality-improvement efforts directed at these patients' care are expected to produce the triple aim of improved health, care experience, and cost-benefit ratio [10, 11]. In this context, the research project *3P, Patients and Professionals in Productive Teams* (2015–2019), had the aim of validating and verifying the prerequisites that support the transformation of a classical profession-centred health care system towards a digitally supported patient-centred service model. The 3P-project has studied service models that were patient-centred, integrated, and proactive in four health organisations located in different regions of Norway and Denmark [12]. The University Hospital of North Norway is one of the included organisations, having an interdisciplinary patient-centred health care team that was run with a cross-organisational service model between the hospital and surrounding municipalities [13]. The aim of the patient-centred health care team was to support the self-management and independent living of elderly patients with chronic diseases and multimorbidities in the hospital discharge transition and during the first weeks at home. The patient-centred service concept was inspired by different care models [14, 15] and aligned with the global strategy on integrated people-centred health services of the World Health Organization (WHO) [16].

In this paper, the existing information flow and digital support of collaborative work within the patient-centred health care team and across organisations has been mapped and evaluated. Based on a qualitative data analysis, several issues were identified that limited the efficiency of the information flow and digital support. To solve those issues, a digital approach is proposed to support the information flow in a more flexible manner for efficient cross-organisational team collaboration within a secure framework. The three research questions (RQs) stated for this study were as follows:

  RQ1: *how can a digital approach support the communication processes and information needs in cross-organisational health care teams*?
  RQ2: *what technical infrastructure can be recommended for a digital approach supporting the information flow in cross-organisational health care teams*?
  RQ3: *what are the benefits and constraints of the digital approach for the information flow in cross-organisational health care teams*?

Following this introduction, the research methodology is described. The results of the explorative study are presented in the next section, together with a proposed set of requirements and functionality for a digital approach. Furthermore, a discussion of the main results is provided, and finally, a summary of the study contribution and conclusions is provided.

## 2. Methodology

Qualitative research methods were used for data collection and analysis [17, 18]. The study was conducted in three phases: (1) June 2017, (2) November 2017, and (3) October 2018, with a total of nine days spent in the health organisation. The recruitment of study participants was made in collaboration with a department manager and 24 informants with multiple professions took part in the study, see Table 1.

### 2.1. The Data Collection

The first phase of the data collection focused on mapping the information flow and digital support of cross-organisational work. Three interviews were made: (1) a focus group with four nurses and the department manager, (2) a semistructured interview with a nurse and physiotherapist pair, and (3) an individual semistructured interview with a physician. A preliminary summary was made of the interviews, and a workshop was organised with the purpose of validation and feedback. 14 informants participated in the workshop, where the identified constraints of the information flow were discussed. The participants were asked to propose and outline an optimal digital support for the information needs in a future perspective. To complete this phase, two technicians were interviewed targeting information and communication technology, and to represent the user perspective, two interviews were made with an elderly patient at home and a family member.

The second phase focused on the functionality of the technology and user experiences. A field study was made with observations of the communication procedures and the technology use in the staff room. Two main technical systems were used, and a thorough demonstration was made of both. Five interviews were made: (1) four semistructured individual ones with nurses and (2) a focus group with four home nurses in a surrounding municipality. The interviews targeted cross-organisational information sharing and collaborative work.

The third phase focused on problem solving, *how to deal with the obstacles in the digital support and optimise the information flow*? A field study was made in the staff room, observing communication and digital support. Five interviews were made: (1) four semistructured individual ones with key informants that had been interviewed in previous phases and (2) a focus group with the same four informants to summarise the insights and for validation purposes. To complete the data collection, an elderly patient was interviewed at home focusing on communication procedures with the team.

### 2.2. Data Analysis

The interviews were audio recorded, in total 13.5 hours. Each session had a duration of 30–120 minutes. Annotations and field notes were made during observations and interviews. The data material was qualitatively analysed and categorised thematically [19], followed by abductive reasoning through a cyclic process. The aim was to describe a best practice for the components and content of importance when designing and implementing digital support systems for person-centred health care services models. The authors have background from health informatics and/or medical practice and share the professional experience of working in clinical environments, and as they have expertise in the actual domain, this represents realism in the proposed set of possible factors and their corresponding detailed description.

### 2.3. Ethical Considerations

The Norwegian Centre for Research Data approved this study with the project number 53771 [20]. All participants received verbal and written information about the project and confidential treatment of their collected data. They were informed that their participation was voluntary, and each participant signed a consent form. Participants were informed that they could withdraw at any time without giving any reason. In that case, their data would be consequently withdrawn and deleted. To minimise the assessment burden, only informant background that was directly relevant to the research question was recorded, such as professional background [21].

## 3. Results

The results are presented and divided into three categories: (1) cross-organisational information and workflow, (2) constraints in digital support, and (3) proposed digital approach for cross-organisational teamwork.

### 3.1. Cross-Organisational Information and Workflow

The patient-centred health care team was interdisciplinary and had cross-organisational employees divided into two locations that were physically placed at hospitals. It was funded jointly by the hospital organisation and surrounding municipalities. The interdisciplinary team had the professions: nurse, physiotherapist, occupational therapist, physician, and pharmacist. There were also administrative and research staff. The team was called upon in two main situations: (1) supporting the early discharge from hospital to home in a subacute context after an emergency hospitalisation and (2) supporting municipal services in diagnosis and treatment planning for elderly individuals at risk of an emergency hospitalisation, while still in a municipal care setting. New referrals were made by municipal services, hospital departments, or general practitioners (GPs). Each referral was registered in electronic health record (EHR) and evaluated by key persons in the interdisciplinary team. For new patients included to the team's services, a startup meeting was organised either at hospital or the patient's home, depending on the patient's whereabouts at the point of referral. Key persons from the interdisciplinary team, municipal services, and optionally family members were present, and the guiding principle was always to start by asking the patient “what matters to you?” and addressing the care supporting the personal long-term goals. Each patient's team had a dynamic organisation, with members included based on the competence needed. A risk analysis was made regarding the patient's situation with prioritisation of critical needs and necessary support. A digital personalised plan with actions was made for each patient.

Figure 1 shows the information and workflow across the actors involved in the patient-centred care process.

### 3.2. Constraints in the Digital Support of Cross-Organisational Teamwork

#### 3.2.1. Tools for Coordination and Planning

There was no e-team support. In the morning meeting, there was a paper-based team book with hand-written actions and plans that was used for the follow-ups of each day. The staff was manually divided into groups and tasks. The telephone was frequently used for information sharing in the cross-organisational teamwork. There were simple and standardised e-messages between the patient-centred team, the GPs, and the municipal home care services. This was a semielectronic solution with secured message exchange between the health care organisations, using ebXML as the syntax for a national eHealth message standard [22–24]. However, the solution only allowed defined documents to be exchanged between the sender in the organisation and the recipient, which was a limitation in situations where ad-hoc access to shared information in the cross-organisational team was needed. When attending patients at home, there was no access to medical information from mobile platforms.

#### 3.2.2. Interoperability and System Integration

Two separate electronic health record systems were used to carry out the services of the patient-centred health care team. The systems had limited interoperability and were administrated and operated by two different organisations. As a consequence, each user had two different login procedures to different desktops, one for each system. For legal obligations, all statutory medical information had to be entered to both systems for permanent data storage, and it was not allowed to transfer text between the systems. Because of that, information was manually entered twice, with the related added workload and was experienced as an inefficient. In the initial phase of the project, temporary permission for cross-organisational electronic health record access was granted, under the quality-improvement project legislation. Such access is normally not allowed under Norwegian regulations, but under evaluation as a permanent solution by the authorities.

#### 3.2.3. Patient and Family Involvement

Patients in the particular health region had reading access to their own hospital electronic health record through the National Health Portal (helsenorge. no), with a secure login procedure. The patient had access to all referrals and progress notes made by different professions, but not to the personalised digital plan and actions. For the municipal electronic health record, the patients had neither GP nor care service access to their own health data. E-consultation was not available and patients had to be attended at home. Medical equipment used by the patients at home for registration of vital signs, telecare alarms, and telemedicine support was standalone solutions and not integrated with the existing systems. There was no technical functionality to involve the family or the network of the patient. The patient interviews revealed that this elderly patient group had a limited digital literacy, a constraint for using technology with complex user interfaces, and secure login with codes and passwords.

### 3.3. Proposed Digital Approach for Cross-Organisational Teamwork

To solve the issue with lacking cross-organisational teamwork support, a new cloud-based portal within the National Health Network is proposed. This would also address the limited integration between the technical systems used in the team-based services.

Automatic data access should be administered from the electronic health record systems of the involved organisations, with login authorisation for the defined users of the interdisciplinary team members. The services of the cloud-based portal would consist of databases for storing necessary data and health care plans, a plurality of team-support functionalities, and a personal workspace for each user.

Such functionalities in the cloud-based portal would extend the use of those services compared to traditional solutions of cloud computing in health care, as they in many cases just provide an internet-/web-based data sharing model [25]. The main benefits on this proposed solution is to place the data storage and team-support functionalities within a neutral domain, independent of the boarders and existing firewalls in the health care organisations. This is beneficial for cross-organisational e-collaborative teamwork.

By establishing access to National Health Registers, advanced search functions can be incorporated in order to identify persons at risk and such risk stratifications are important for initiating proactive services.

Patients should also be users of the proposed cloud-based solution. Patients in Norway have a statutory right to access their health data and some can already approach several health services and have digital reading access to personal health information in the National Health Portal (helsenorge. no). However, within the proposed solution, the objective is to enable empowerment of the patient, with self-management functions such as measurements of vital signs parameters and recording of disease-specific symptom scores that may impact on medical decision-making. The individual plan “what matters to the person?” should be stored and maintained in the portal, both by the patient and professionals. An e-consultation function would open for electronic communication between the patient, family members, and health care professionals.

Figure 2 describes the proposed cloud-based health portal to solve limitations in the cross-organisational team-based work and information flow.

Table 2 presents the proposed requirements and functionalities for the cloud-based portal described in Figure 2.

## 4. Discussion

This paper has presented a study on the digital support in an interdisciplinary and cross-organisational patient-centred health care team. The aim was to identify challenges in the information flow, evaluate the technology in use, and propose an improved solution. The study showed that there were several limitations and constraints in the technology that impacted on the clinical routines and the workflow of the patient-centred health care team. The three research questions (RQs) formulated at the beginning of this paper are answered below based on the results from the study.

The RQ1 asked about how a digital approach can support the information flow in cross-organisational care teams. The study showed that the existing technologies had shortcomings in the support of teamwork functionality, also seen in [26]. There was a need for tools to support coordination and planning within the patient-centred health care team and across organisations. To make this easier, the user-friendly integration [27, 28] into a cloud-based combined workspace will be of importance, with automatic back-end synchronizing of stored information to the relevant electronic health record systems. The administrative tasks and involving team members with necessary competence should be managed by the team coordinator. For communication with other health care providers such as GP or municipal services, instead of using the telephone, the cloud-based solution would support fast exchange of information, but also task handling functions for confirming that information was received and action was taken, in line with [29]. Other support functions are real-time information of health care action plans and use of mobile devices to access this information at the point-of-care.

The RQ2 asked about a recommended technical infrastructure for the digital approach. In the study, it was confirmed that the lacking interoperability and limited integration between the existing systems because of legal challenges caused additional workload in the cross-organisational workflow, similar to [30]. To solve the digital constraints, the proposed cloud-based health portal should be hosted in the National Health Network security service [22] with automatic data access between the electronic health record systems of the involved organisations. There should be a database for storing of data and digital health care plans, together with team-support functionalities. Each team member should have a digital personal workspace within the portal for overview of tasks, actions, and progress. Functions for e-support and two-way virtual meetings, also with the patient and/or close relatives, should be incorporated, in line with [28]. Integration of telecare alarm systems and telemedicine technology can be of important value for the patient; however, such solutions are normally implemented in different silo functions and not connected to the defined personal care plan and the team support and follow up, which can cause misunderstandings and fragmented patient support, also described in [31].

The RQ3 targeted the benefits and constraints of the proposed digital approach. The cloud-based health portal with a shared workspace and teamwork functionality would support the information flow and ease the access to important information to all the members of the team and collaborating health providers across organisations. The risk stratification function is beneficial and important for the provision of proactive services, in line with [32, 33], requiring the capabilities of combining advanced search functions between different electronic health record systems and national health registers. However, a user-friendly integration of such functions is of high importance because of multiple-user groups and the complexity in defining adequate parameters to define patients at risk [28].

Constraints might be the challenges, both legally for cross-organisational shared access to health records across the different domains involved and information security precautions for authorisation of the actual persons within each patient's follow-up team. New experts need to be incorporated on ad-hock basis depending on the patient's actual situation, which might differ. Such flexibilities represent both organisational and technical challenges. In addition, there is a cost of the system construction, network infrastructure, user interface design, and back-end management. Also, the liability in developing and providing new shared solutions for the patient's reading and writing access to the cloud-based health portal is an unclear situation as health care organisations normally limit their obligations to initiatives within their own domain, and national governmental initiatives could be the future action and platform hosting such solutions [34]. Private initiatives and proprietary cloud services are today targeting the consumer market with new health and care solutions. This paradigm should be addressed in future studies.

This study had some limitations such as studying the service model for a cross-organisational patient-centred care team in only one health region. However, the respectable number of study participants with different professions and backgrounds meaningfully represented the group and contributed to the study in multiple settings, reflecting the general situation in Norway. The research method, combining qualitative analysis with abductive reasoning, provided insights into the research team regarding benefits and barriers of both existing and proposed new digital solutions.

## 5. Conclusions

This study with an evaluation of digital support was made as a part of the research project *3P*, *Patients and Professionals in Productive Teams*, which aimed to evaluate models for patient-centred cross-organisational health care teams. The explorative evaluation showed a lacking interoperability between the digital systems and a limited support for cross-organisational teamwork, causing raised manual efforts to maintain the information flow. The main implications of this study are the proposed principles for a cloud-based health portal with a shared workspace and teamwork functionality for cross-organisational health care teams. Those principles are transferable to a multitude of clinical contexts where ad-hoc based access to shared medical information is of importance for decision-making and life-saving treatment. The next step will be development of a user interface and necessary software programming in order to develop a pilot to be used in a user evaluation study, before system implementation for daily routine use in the health care sector. The results presented are in line with and reflect on national strategies in Norway focusing on primary health care teams with implemented e-consultation and video facilities [35]. However, the need of flexible information flow and teamwork functionalities as proposed in this paper is yet not fully exposed and should define a fundamental basis for innovative experiments for new health care services of the future [36].

In terms of future work, it is suggested to address further research on other patient-centred cross-organisational settings using interoperable information cloud and focusing on the hosting and governing of it, and the information sharing across different platforms.

## Figures and Tables

**Figure 1:** The information flow cycles in the interdisciplinary team across organisations: (1) e-messages of a new patient from the hospital to team coordinator. (2) Visit to the patient while in hospital. (3) Discuss the actual patient problems in an interdisciplinary team meeting. (4) Team meeting and analysis of risk factors. (5) Define a digital personalised plan with actions. (6) The digital personalised plan with actions is documented in both the hospital's EHR and the municipality's EHR systems. (7) The patient is discharged from the hospital with home care follow-up. (8) Information e-message sent to the local doctor (GP). (9) Information e-message sent to the municipality home care service. (10) An interdisciplinary health and care team support is established to follow up planned actions (mean 30 days). (11) On-going activity and reports documented in the hospital's EHR and in the municipality's EHR systems. (12) Handover of care plan to municipal home care services for regular visits at home.

**Figure 2:** The cloud-based health portal. The workflow functionalities can be obtained: (1) Notification of a new patient can be sent from the hospital to the team coordinator. (2) Normally, the team coordinator will need to meet the patient while at hospital or at home to define the needs and wishes for the patient. (3) Team members and their access can be defined by the team coordinator. (4) In a virtual team meeting, risk factors can be identified. (5) All information collected and defined health care plans with actions are shared between all interdisciplinary team members, and also with the patient and/or close relatives. (6) The patient can access all information and can be notified of action points. (7) Automated data transfer needs to be established from the patient's vital sign devices, including questionnaires and patient-reported outcome reports. (8) Automatic access from the local doctor's EHR system to the cloud portal with notifications. (9) Automatic access from the municipality's EHR system to the cloud portal with notifications. (10) An interdisciplinary health and care team support is established to follow up planned actions (mean 30 days). (11) On-going activity and reports documented in the cloud portal. (12) Handover of care plan to municipal home care services for regular visits at home.

**Table 1:** Distribution of the participants' profession.

Profession	*n* = 24
Physician	1
Nurse	13
Physiotherapist	1
Occupational therapist	1
Administrator	3
Technician	2
Patient	2
Family member	1

**Table 2:** The requirements for the cloud-based health portal.

*Shared cloud portal*
Define a shared collaborative workspace, with secure access from actual health care team members and the patient/close relatives, based on regulations for privacy and security.
Implement cross-organisational access from the patient's electronic health record to all the involved systems (hospital, local doctor/GP, municipality home care services, and national health portals with relevant information and functions).
A customised workspace and user interface on all relevant platforms, also for mobile solutions.
Automatic back-end synchronizing of stored information to the relevant EHR systems (at the hospital, local doctor/GP, municipality home care services) for necessary medical documentation and activity log documentations.

*Information flow functionalities*
Integrated information flow, where all team members involved have immediate access to relevant real-time information and current patient status.
Real-time information of health care action plans and status of tasks, with two-way e-communication between team members and the patient.
Constant visualization in a dashboard of defined risk factors, risk stratification, and the progress.
Health care actions and support with visual indication of fulfilment and improvements according to a plan.
Automatic trigger of unexpected events or unnormal deviations according to a plan, based on triage algorithms.
Integration of electronic prescriptions to keep control of active medications, also integrated with a patient's medicine dispenser with programmed time intervals to monitor medication taken and with relevant warnings.

*Patient involvement and support*
Registration of «what I want my carers to know about me?» and «what matters to me?»
Integration of telemedicine functions with the patient's self-monitoring and recording of vital sign parameters with regular report on status based on disease-specific questionnaires and patient-reported outcomes reports.
Integration with implanted devices and sensors such as pacemakers and ICD systems that regularly report cardiac situations and arrhythmia events. Blood glucose sensors that monitor and regulate insulin therapy.
Integration with medical equipment used by the patient such as PAP/CPAP/sleep apnea assistance technology, home respiration equipment, and home dialysing equipment.
Implemented e-consultation functionalities with video solutions in order to facilitate virtual contacts and remote medical consultations.
Implement virtual rehabilitation plans and activities for the patient to self-manage and carry out defined activities for training and re-establish functions for active daily living.
Electronic messages and support for the patient in a user-friendly workspace with easy access to all relevant information and personal activity tasks.
Integration of mobile self-help and well-being third-party applications.

*Teamwork support*
Teamwork functionality with easy involvement of new team members for the particular patient depending on the actual situation and competence needed.
Task handling function, where a dedicated task can be assigned to a specific person for follow-up within a deadline, and a visual overview for all team members on the ongoing tasks with status.
The patient's own daily tasks and recordings of activity and medical measurements are automatically included in a visual dashboard showing the degree of self-management and improvements according to a plan.
Integration of telecare alarm systems and response centre services for necessary actions and follow-up on critical alarms and warnings.

## Data Availability

The recorded data used to support the findings of this study have not been made available because of national regulations regarding the privacy of the study participants.
